# Association between Genetic Polymorphisms in Methylenetetrahydrofolate Reductase and Risk of Autoimmune Diseases: A Systematic Review and Meta-Analysis

**DOI:** 10.1155/2022/4568145

**Published:** 2022-05-31

**Authors:** Mao Lu, Ke Peng, Li Song, Li Luo, Peng Liang, Yundan Liang

**Affiliations:** ^1^Department of Dermatovenereology, The First Affiliated Hospital of Chengdu Medical College, Chengdu, Sichuan 610500, China; ^2^School of Clinical Medicine, Chengdu Medical College, Chengdu, Sichuan 610500, China; ^3^Department of Pathology and Pathophysiology, School of Basic Medical Sciences, Chengdu Medical College, Chengdu, Sichuan 610500, China

## Abstract

Methylenetetrahydrofolate reductase (MTHFR) is a critical rate-limiting enzyme in the homocysteine/methionine metabolism pathway that is implicated in the pathogenesis and progression of autoimmune diseases. Previous association studies have been performed to investigate the effect of polymorphisms in *MTHFR* on the risk of autoimmune diseases with inconsistent results. Therefore, this meta-analysis was designed to assess the association between the *MTHFR* 677 C/T and 1298 A/C polymorphisms and the susceptibility to autoimmune diseases. We identified reports by a literature search in the following electronic databases: PubMed, Ovid, Web of science, and China National Knowledge Infrastructure. Statistical analyses of the summary odds ratios (ORs) and 95% confidence intervals (CIs) were done using STATA software. In a recessive genetic model, the *MTHFR* 677 C/T polymorphism was associated with an increased risk of Behcet's disease (OR = 1.97, 95% CI, 1.31-2.97), multiple sclerosis (OR = 1.57, 95% CI, 1.03-2.38), and ankylosing spondylitis (OR = 2.90, 95% CI, 1.92-4.38). The *MTHFR* 1298 A/C polymorphism was associated an increased risk of multiple sclerosis in a heterozygote comparison (OR = 2.36, 95% CI, 1.29-4.30) and in a dominant model (OR = 2.31, 95% CI, 1.24-4.29). This meta-analysis demonstrated that the *MTHFR* 677 C/T was a risk factor for Behcet's disease, multiple sclerosis, and ankylosing spondylitis, and the 1298 A/C was a risk factor for multiple sclerosis.

## 1. Introductions

Autoimmune diseases are a group of diseases characterized by abnormal immune response to autoantigens and self-tissue destruction [1, 2]. It is estimated that 7.6-9.4% of global population is affected by autoimmune diseases, causing the cost of treatment great than 100 billion annually [3, 4]. Despite the high price of treatment, autoimmune diseases cannot be cured but only temporarily reduce symptoms. The major reason for the therapeutic problem may be that the exact mechanism of triggering the disease is not yet fully known. A previous work has demonstrated that environmental exposure may help individuals with a genetic predisposition to develop autoimmune diseases, suggesting the combination of genetic and environmental factors may contribute to the risk of the disorder [5, 6].

Increasing evidence has shown that abnormal metabolism of folate and homocysteine is involved in the pathogenesis of autoimmune diseases [7, 8]. Homocysteine (Hcy), first discovered in 1969, is a nonproteinogenic *α*-amino acid that is an intermediary product in methionine metabolism [9]. Elevated levels of total Hcy were observed in some autoimmune diseases, such as psoriasis [10], multiple sclerosis (MS) [11], Behcet's disease (BD) [12], ankylosing spondylitis (AS) [13, 14], and Graves' disease (GD) [15]. A critical rate-limiting enzyme in Hcy/methionine metabolism is methylenetetrahydrofolate reductase (MTHFR). Several mutations of the gene coding the MTHFR enzyme, such as the substitution of proline to leucine, threonine to methionine, and alanine to valine were found to be associated with low activity of MTHFR, resulting in impaired folate metabolism and accumulation of Hcy [16, 17].

*MTHFR*, located on the long arm of chromosome 1 (chr1p36.3) in humans, contains several missense mutations that caused altered amino acid in the protein product. Among them, rs1801133 (677 C/T) and rs1801131 (1298 A/C) were studied widely [18]. The rs1801133 consists of a transition of C to T at the residue 677, leading to an alanine to valine substitution and the rs1801131 consists of a transition of A to C at the nucleotide position 1298, leading to a glutamate to alanine substitution. Both the single-nucleotide polymorphisms (SNPs) were related to the reduction of MTHFR enzymatic activity and higher levels of Hcy [19–23]. The MTHFR, catalyzing the synthesis of 5-methyltetrahydrofolate, is required for vitamin B12-dependent enzyme methionine synthase and Hcy regulation [24, 25]. Vitamin B12 deficiency and Hcy imbalance have been identified to play a role in the pathology of psoriasis [26], MS [27], BD [28], AS [29], and GD [30]. Previously, some authors reported that the two genetic variants were risk factors for psoriasis [31], MS [32], and GD [33]. Not all reports, however, supported these findings. For example, Chorąży et al. reported that there was no statistically significant association between the *MTHFR* 677 C/T and 1298 A/C polymorphisms and MS risk [34]. The conflict results might be caused by inadequate statistical power, ethnic diversities, and publication bias. In this meta-analysis, we aimed to evaluate the association between the *MTHFR* 677 C/T and 1298 A/C polymorphisms with the susceptibility of autoimmune diseases, including psoriasis, MS, BD, AS, and GD.

## 2. Materials and Methods

### 2.1. Search Strategy

The systematic review and meta-analysis followed the PRISMA 2020 statement guideline [35]. Reports investigating the association of *MTHFR* polymorphisms with autoimmune diseases, including psoriasis, BD, GD, AS, and MS were identified before July 2021. The literature search was performed in the following electronic databases: PubMed, Ovid, Web of science, and China National Knowledge Infrastructure. The following items were used: “methylenetetrahydrofolate reductase”, “MTHFR”, “polymorphism”, “variant”, “SNP”, “psoriasis”, “Behcet's disease”, “Graves' disease”, “ankylosing spondylitis”, and “multiple sclerosis”. Additional articles were retrieved by checking references that were cited in the selected articles. No language restrictions were applied for the search strategy.

### 2.2. Inclusion and Exclusion Criteria

We included case-control and case-cohort studies that investigated the association of the *MTHFR* 677 C/T or 1298 A/C polymorphism with the following autoimmune diseases, including psoriasis, BD, GD, AS, and MS. We excluded studies that were case report, review articles, and records with insufficient data for calculating odds ratio (OR) and 95% confidence interval (CI). Studies that presented overlapping cases or controls were also excluded.

### 2.3. Data Extraction

LM and PK reviewed and extracted simultaneously the data using a predefined form. The following information was extracted: the first author's name, year of publication, country of origin, ethnicity, sample size, definition of cases and controls, genotyping technique, and quality control of genotyping technique. Interreviewer disagreements were resolved by discussion with the third author (LY) who double checked the raw data.

### 2.4. Assessment of Study Quality

With reference to the Newcastle-Ottawa Scale, we assessed the quality of included studies by dividing them into two groups: high-quality (equal or more than 4 stars) and low- quality (less than 4 stars) studies. The assessment was performed independently by LM and PK, and discrepancies were resolved by consultation with LY.

### 2.5. Statistical Analysis

Hardy-Weinberg equilibrium (HWE) was assessed using a chi-squared test. The *Q*-statistic test and *I*^2^ metric were used to assess the heterogeneity across studies [36]. If the *P* value was more than 0.10 and *I*^2^ was less than 50%, indicating that there was no heterogeneity, the fixed-effect model was used; otherwise, the random-effect model was used [37, 38]. To compare the association between *MTHFR* polymorphisms and the risk of autoimmune diseases, four comparisons (i.e., heterozygote, homozygote, dominant, and recessive genetic models) were used by computing summary OR and 95% CI. Subgroup analyses based on racial decent (Asians and Caucasians) and study quality were also done. The robustness of results was evaluated using a sensitivity analysis when removing a single study at a time. Egger's linear regression asymmetry test was used to assess publication bias of included studies [39]. A two-tailed *P* value < 0.05 was considered significant. All the statistical analyses were performed using STATA software version 11.0 (Stata Corporation, College Station, TX).

### 2.6. Trial Sequential Analysis

Trial sequential analysis (TSA) software version 0.9.5.10 beta was used to assess the reliability of the results from meta-analysis [40]. The O'Brien-Fleming boundary, futility boundary, and *Z*-curve were constructed with a type I error of 5%, power of 80%, and relative risk reduction of 5-20%. Required information size (RIS) was also estimated. For the *MTHFR* 677 C/T polymorphism, TSA was performed under a recessive genetic model; for the 1298 A/C polymorphism, TSA was performed under a dominant genetic model.

## 3. Results

### 3.1. Eligible Studies

The literature review identified 262 citations. After duplicating removing, 161 appeared to be relevant to the meta-analysis and were selected for further analysis. Among them, 78 were excluded after review of title and abstract. The full texts of the remained studies were read, and 40 were excluded due to different reasons, such as no *MTHFR* polymorphisms, lack of autoimmune diseases, absence of controls and available data, review articles, overlapping data, and case report. Finally, 43 studies met the inclusion criteria and were enrolled in the meta-analysis, including 14 investigating psoriasis, 10 investigating BD, 9 investigating MS, 5 investigating AS, and 3 investigating GD (Figure 1).

Detailed characteristics extracted from the eligible studies are summarized in Table 1. Of the 43 included studies, 15 were carried out in Asians and 28 were carried out in Caucasians. Publication date ranged 1997–2020 and the number of sample sizes ranged 60–844. In summary, less than 40% (17/43) records were perceived as high-quality studies and more than 90% (40/43) studies were in agreement with HWE.

### 3.2. Association of *MTHFR* Polymorphisms with Psoriasis Risk

Fourteen studies investigated the association of the *MTHFR* 677 C/T polymorphism with psoriasis risk, involving 2351 cases and 2421 controls (Figure 2). Meta-analysis showed a borderline statistical significance between the *MTHFR* 677 TT genotype and the presence of psoriasis in overall analysis (OR = 1.57, 95% CI, 1.00-2.45). The borderline statistical significance was also observed in Caucasians (CT vs. CC: OR = 1.93, 95% CI, 1.01-3.69; CT/TT vs. CC: OR = 2.06, 95% CI, 1.04-4.05, respectively) rather than in Asians. In subgroup analysis based on study quality, no significant association of the *MTHFR* 677 C/T polymorphism with psoriasis risk was found in both high-quality and low-quality studies (Table 2). Sensitivity analysis revealed that the exclusion of the study by Izmirli et al., Luo et al., or Wang et al. yielded a different result for the association of the *MTHFR* 677 C/T polymorphism with psoriasis risk [41–43].

Five studies investigated the association of the *MTHFR* 1298 A/C polymorphism with psoriasis risk, involving 862 cases and 1024 controls (Table 3, Figure 3). Two studies were carried out in Asians, and 3 studies were carried out in Caucasians. A significant association was found between the *MTHFR* 1298 CC genotype and the presence of psoriasis in Asians (CC vs. AA: OR = 3.25, 95% CI, 1.68-6.31; CC vs. AA/AC: OR = 2.68, 95% CI, 1.39-5.16, respectively). In overall analysis, no significant association of the *MTHFR* 1298 A/C polymorphism with psoriasis risk was found. In sensitivity analysis, however, the exclusion of the study by Agha et al., Beranek et al., or Wu et al. yielded a significant result [44–46].

### 3.3. Association of *MTHFR* Polymorphisms with BD Risk

Ten studies investigated the association of the *MTHFR* 677 C/T polymorphism with BD risk, involving 825 cases and 892 controls (Figure 2). Among them, 9 were performed in Caucasians. Meta-analysis showed a statistical significance between the *MTHFR* 677 TT genotype and the presence of BD in overall analysis (TT vs. CC: OR = 2.00, 95% CI, 1.30-3.07; TT vs. CT/CC: OR = 1.97, 95% CI, 1.31-2.97, respectively) and Caucasians (TT vs. CT/CC: OR = 1.84, 95% CI, 1.19-2.86). After subgroup analysis based on study quality, the significant association of the *MTHFR* 677 C/T polymorphism with BD risk was also found in low-quality studies (TT vs. CT/CC: OR = 1.62, 95% CI, 1.03-2.54) (Table 2). Sensitivity analysis revealed that the exclusion of the study by Karakus et al. generated a nonsignificant result for the association of the *MTHFR* 677 C/T polymorphism with BD risk [47].

### 3.4. Association of *MTHFR* Polymorphisms with MS Risk

Nine studies investigated the association of the *MTHFR* 677 C/T polymorphism with MS risk, involving 1227 cases and 1426 controls (Figure 2). Meta-analysis showed a borderline statistical significance between the polymorphism and the presence of MS in a recessive genetic model (OR = 1.57, 95% CI, 1.03-2.38). In subgroup analysis based on study quality, the borderline significant association of the *MTHFR* 677 C/T polymorphism with MS risk was also found in low-quality studies (TT vs. CC: OR = 2.18, 95% CI, 1.04-4.55; TT vs. CT/CC: OR = 2.21, 95% CI, 1.53-3.19, respectively) (Table 2).

Seven studies investigated the association of the *MTHFR* 1298 A/C polymorphism with MS risk, involving 952 cases and 1232 controls (Table 3, Figure 3). All the studies were conducted in Caucasians. Meta-analysis showed a statistical significance between the *MTHFR* 1298 A/C polymorphism and the presence of MS in overall analysis (AC vs. AA: OR = 2.36, 95% CI, 1.29-4.30; AC/CC vs. AA: OR = 2.31, 95% CI, 1.24-4.29, respectively) and subgroup analysis, such as high-quality studies (AC vs. AA: OR = 4.64, 95% CI, 1.08-19.88) and low-quality studies (AC vs. AA: OR = 1.50, 95% CI, 1.05-2.15; AC/CC vs. AA: OR = 1.50, 95% CI, 1.09-2.07, respectively) (Table 3). Sensitivity analysis revealed that the exclusion of an individual study at a time did not change the findings of the *MTHFR* 677 C/T and 1298 A/C polymorphisms increasing MS risk.

### 3.5. Association of *MTHFR* Polymorphisms with as Risk

Five studies investigated the association of the *MTHFR* 677 C/T polymorphism with AS risk, involving 545 cases and 502 controls (Figure 2). Among them, 3 were performed in Asians and 2 were performed in Caucasians. Meta-analysis showed a statistical significance between the *MTHFR* 677 C/T polymorphism and the presence of AS in overall analysis (TT vs. CC: OR = 3.09, 95% CI, 1.99-4.80; CT/TT vs. CC: OR = 1.33, 95% CI, 1.04-1.72; TT vs. CT/CC: OR = 2.90, 95% CI, 1.92-4.38, respectively). In subgroup analysis, the significant association of the *MTHFR* 677 C/T polymorphism with MS risk was also found in Asians (TT vs. CC: OR = 2.91, 95% CI, 1.82-4.65; CT/TT vs. CC: OR = 1.60, 95% CI, 1.16-2.19; TT vs. CT/CC: OR =2.67, 95% CI, 1.73-4.14, respectively), Caucasians (TT vs. CC: OR = 4.55, 95% CI, 1.27-16.27; TT vs. CT/CC: OR = 5.14, 95% CI, 1.44-18.33, respectively), high-quality studies (TT vs. CC: OR = 2.61, 95% CI, 1.42-4.82; TT vs. CT/CC: OR = 2.48, 95% CI, 1.42-4.32, respectively), and low-quality studies (TT vs. CC: OR = 3.65, 95% CI, 1.94-6.90; CT/TT vs. CC: OR = 1.72, 95% CI, 1.16-2.53; TT vs. CT/CC: OR = 3.45, 95% CI, 1.86-6.42, respectively) (Table 2). Sensitivity analysis showed that the result was not affected when excluding a single study each time.

### 3.6. Association of *MTHFR* Polymorphisms with GD Risk

Three studies investigated the association of the *MTHFR* 677 C/T and 1298 A/C polymorphisms with GD risk (Tables 2 and 3, Figures 2 and 3). All the studies were conducted in Asians. No statistical significance between the *MTHFR* 677 C/T and 1298 A/C polymorphisms and the presence of GD were observed. Sensitivity analysis showed that the result was not changed when excluding a single study each time.

### 3.7. TSA Analysis

The cumulative Z-curve in Figure 4(a) crossed the futility boundary and the RIS boundary, indicating that it is unnecessary for additional studies to investigate the association between the *MTHFR* 677 C/T and psoriasis risk. The cumulative *Z*-curve in Figures 4(b)–4(d) and 4(f) crossed the traditional boundary and the O'Brien-Fleming boundary, indicating that the results from the meta-analysis may be conclusive. However, the cumulative *Z*-curve in Figures 4(e), 4(g), and 4(h) did not cross any boundary, indicating that the findings of the *MTHFR* 1298 A/C with psoriasis risk and the 677 C/T and 1298 A/C with GD risk are inconclusive.

### 3.8. Heterogeneity Analysis and Publication Bias

During pooled analysis of *MTHFR* 677 C/T and 1298 A/C polymorphisms with psoriasis and MS risk, the between-study heterogeneity was found. Metaregression was then used to analyze whether some factors such as sample size, ethnicity, HWE, and study quality affected the source of between-study heterogeneity. None of these factors, however, influenced the heterogeneity. Publication bias was evaluated using Egger's linear regression asymmetry test, and no evidence of publication bias was found (*P* > 0.05) (Figure 5).

## 4. Discussion

Autoimmune disease is a pathological state that occurs when self- or autoantigens are misidentified as foreign entities by the immune system, resulting in tissue destruction and chronic inflammation [1, 2]. Although it is unknown exactly what triggers the disturbance of the immune system, there are several predisposing and precipitating factors, such as genetic and environmental factors [5, 6]. As one of the most frequent types of DNA sequence variation in the human genome, SNPs play an important role in individuals' susceptibility to autoimmune diseases [48, 49]. Previous genetic association studies have demonstrated that autoimmune diseases may share a common genetic background [49].

MTHFR is a crucial enzyme in Hcy/folate metabolism, and the *MTHFR* deficiency is related to the development and progression of autoimmune diseases [16, 17]. Previously, two important polymorphisms 677 C/T and 1298 A/C in *MTHFR* were considered to contribute to the occurrence of autoimmune diseases [31–33]. The results, however, are contradictory to the findings from other authors. For example, Asefi et al. reported that the *MTHFR* 677 T allele was associated with an increased risk of psoriasis [50], whereas Beranek et al. failed to find any association between the SNP and risk of psoriasis [45]. Two previous meta-analyses were conducted, and no significant association of the *MTHFR* 677 C/T with the etiology of psoriasis was found [51, 52]. It is necessary to update the data as many more studies appeared during the past years [31, 42, 44, 45, 53]. In this meta-analysis, we did not find any relationship of the SNP with psoriasis in overall comparison. TSA confirmed this finding. Nevertheless, subgroup analyses showed that the association was a borderline statistical significance in Caucasians. Further investigations are of great importance to exclude the possibility of the results occurring by chance.

Apart from psoriasis, the *MTHFR* 677 C/T has been examined extensively whether it influences individuals' susceptibility to BD and MS. However, conflicting results were also obtained. Karakus et al. and Naghibalhossaini et al. reported that subjects carrying the 677 T allele had an increased susceptibility to BD and MS [32, 47], whereas Chorąży et al. and Koubaa et al. reported that the *MTHFR* 677 C/T was not a risk factor for BD and MS [34, 54]. The negative results were verified by subsequent meta-analysis [48, 55]. However, in this updated meta-analysis involving 825 BD cases (892 controls) and 1227 MS cases (1426 controls), we found that the *MTHFR* 677 TT genotype was associated with a higher risk of BD and MS. The discordant results may be due to small sample sizes in the meta-analysis reported by Chamorro et al. that included 494 BD patients and 374 controls [48], and the meta-analysis reported by Lee et al. that included 830 MS patients and 893 controls [55].

Regarding the association between the *MTHFR* 677 C/T and AS risk, 5 studies were included in this meta-analysis. The pooled analysis showed a significant association between AS and the *MTHFR* 677 TT genotype in overall comparison. Subgroup analyses based on ethnicity and study quality also showed the significant association. Notably, carriers with the *MTHFR* 677 TT genotype had a 2.48-increased risk of AS risk in high-quality studies under a recessive genetic model. To the best of our knowledge, this is the first meta-analysis to assess the effect of the *MTHFR* 677 C/T polymorphism on AS risk, which provides stronger evidence than any previous case-control study.

To date, only 3 studies investigated the association between the *MTHFR* 677 C/T and GD risk. When we pooled all data together, only 409 cases and 418 controls were included in the current meta-analysis. TSA also showed that the findings may be not conclusive, and thus, the negative results in the current study should be interpreted with caution. Additional studies are needed to be performed to clarify the exact role of the *MTHFR* 677 C/T in the pathogenesis of GD.

Besides the *MTHFR* 677 C/T, the 1298 A/C polymorphism was reported to be associated significantly with MS risk [56–58]. However, Chorąży et al. did not find any link between the 1298 A/C polymorphism and MS risk [34]. A meta-analysis including 3 studies was performed in 2015, and no association between the *MTHFR* 1298 A/C polymorphism and MS was found [55]. In the present meta-analysis, we enrolled additional studies [32, 34, 56, 59] and found that the *MTHFR* 1298 AC and AC/CC genotypes were associated with increased risks of MS both in overall comparison and subgroup analysis according to study quality. Sample size is an important issue for a sound association study because small samples may result in insufficient power to obtain the real effect. Our study has more samples than previous meta-analysis reported by Lee et al. [55], indicating that we provided more statistical power and stronger evidence to support the positive findings in this study.

The *MTHFR* 1298 A/C polymorphism was also analyzed in psoriasis and GD patients. Not surprisingly, inconsistent results were also observed. Kilic et al. reported that the prevalence of the 1298 C allele was higher by 17.0-fold in patients with psoriasis compared to the control group [31], whereas Luo et al. reported that the genotype distribution of the 1298 A/C was not different significantly between psoriasis patients and controls [42]. In this meta-analysis, although a significantly increased association of the CC and AC/CC genotypes was observed in Asians, there was no significant relationship between the 1298 A/C and psoriasis risk in overall analysis and Caucasians. As only 2 studies were conducted in Asians, the positive results might not be robust enough. When analyzing the association between the *MTHFR* 1298 A/C polymorphism and GD risk, only 3 studies were included in this meta-analysis and no significant association was observed. According to the data from TSA, however, we cannot conclude that the 1298 A/C was not a risk factor for GD since the limited samples may lead to false negative error.

In this meta-analysis, heterogeneity across studies was observed in some comparisons. Unfortunately, we did not identify what caused the heterogeneity. Despite the disadvantages, no publication bias is present, suggesting there is no evidence of publication selection bias in the literature.

This study contains some limitations that should be discussed. The association of the *MTHFR* 677 C/T with psoriasis was borderline significant. After the exclusion of the study by Izmirli et al., Luo et al., or Wang et al., the findings were changed [41–43], suggesting that heterogeneity among studies might affect the result. However, the possible reason for explaining the heterogeneity was not identified. Furthermore, the relationship between the *MTHFR* 677 C/T and 1298 A/C polymorphisms and GD risk was investigated only in a few studies [33, 60, 61]; thus, we were unable to perform stratification analysis by ethnicity. Although we pooled all data from observational studies together, the sample size is still moderate, especially in subgroup analyses, which may lead to lower power for providing strong evidence of the effect of SNPs in *MTHFR* on the risk of autoimmune diseases.

In conclusion, this meta-analysis demonstrated that the *MTHFR* 677 C/T was a risk factor for BD, MS, and AS and the 1298 A/C was a risk factor for MS. Considering the small number of studies included in some certain subgroups, further larger-sample investigations performed in diverse ethnic groups are necessary to confirm these findings. Functional analyses are also required to elucidate whether and how the SNPs in *MTHFR* impact the etiology of autoimmune diseases.

## Figures and Tables

**Figure 1:** Flow diagram of selection studies.

**Figure 2:** Forest plots of *MTHFR* 677 C/T with the risk of psoriasis (a), Behcet's disease (b), multiple sclerosis (c), ankylosing spondylitis (d), and Graves' disease (e).

**Figure 3:** Forest plots of *MTHFR* 1298 A/C with the risk of multiple sclerosis (a), psoriasis (b), and Graves' disease (c).

**Figure 4:** Trial sequential analysis of the association between *MTHFR* 677 C/T and the risk of psoriasis (a), Behcet's disease (b), multiple sclerosis (c), ankylosing spondylitis (d), and Graves' disease (e) under a recessive model. Trial sequential analysis of the association between *MTHFR* 1298 A/C and the risk of multiple sclerosis (f), psoriasis (g), and Graves' disease (h) under a dominant model.

**Figure 5:** Egger's funnel plot for evaluating publication bias of *MTHFR* 677 C/T with the risk of psoriasis (a–d) and Behcet's disease (e–h). (a, e) 667CT vs. CC. (b, f) 667TT vs. CC. (c, g) 667CT/TT vs. CC. (d, h) 667TT vs. CC/CT.

**Table 1:** Characteristics of literatures included in the meta-analysis.

First author	Year	Country	Ethnicity	Diagnosis of cases	Controls	Number of cases/controls	Matching criteria	Genotyping method	Quality control	Polymorphisms	Newcastle-Ottawa scale	Diseases
Agha	2018	Pakistan	Caucasian	—	Adults unrelated to cases and without a history of psoriasis	200/200	—	PCR-RFLP	—	677 C/T; 1298 A/C	★★	Psoriasis
Alatab	2011	Iran	Caucasian	According to the McDonald criteria	Healthy volunteers	194/230	Age and sex	PCR-RFLP	DNA sequencing.	677 C/T	★★★★★	MS
Arakawa	2012	Japan	Asian	According to a clinical history of thyrotoxicosis and a positive test for anti-thyrotrophin receptor antibody	Healthy volunteers	160/83	—	PCR-RFLP	—	677 C/T; 1298 A/C	★★★	GD
Asefi	2014	Iran	Caucasian	Psoriasis area and severity index	Healthy subjects	100/100	Age, gender, and race	DNA sequencing	Genotyping was performed without knowledge of cases and controls.	677 C/T	★★★★★	Psoriasis
Beranek	2019	Czech Republic	Caucasian	—	Healthy subjects	35/60	—	TaqMan	—	677 C/T; 1298 A/C	★★	Psoriasis
Bin	2019	Saudi Arabia	Caucasian	Plaque psoriasis for at least 1 year	Healthy subjects	106/280	Age and sex	PCR-RFLP	Positive, negative control and repeated genotyping were used.	677 C/T	★★★★	Psoriasis
Cakina	2019	Turkey	Caucasian	According to the McDonald criteria	Healthy subjects	80/80	Age and sex	PCR-RFLP	—	677 C/T; 1298 A/C	★★★	MS
Canataroglu	2003	Turkey	Caucasian	The criteria of the International Study Group for BD	Healthy subjects	40/60	—	Light Cycler real-time PCR	—	677 C/T	★★★	BD
Caramaschi	2010	Italy	Caucasian	The criteria of the International Study Group for BD	Healthy subjects	30/30	—	PCR-allele specific oligonucleotide	—	677 C/T; 1298 A/C	★★★★	BD
Cevik	2014	Turkey	Caucasian	According to the 2005 Revised McDonald MS criteria	Healthy subjects	130/150	Age and sex	PCR-RFLP	—	677 C/T	★★★★★	MS
Chorąży	2019	Poland	Caucasian	According to the McDonald criteria	Healthy volunteers without a family history of any autoimmune disease	174/186	—	TaqMan	—	677 C/T; 1298 A/C	★★★	MS
Dashti	2020	Kuwait	Caucasian	—	Healthy volunteers	170/311	Age and sex	TaqMan	—	1298 A/C	★★★	MS
Espinosa	2002	Spain	Caucasian	The criteria of the International Study Group for BD	Healthy subjects	38/100	—	PCR-RFLP	—	677 C/T	★★★★	BD
Fekih Mrissa	2013	Tunisia	Caucasian	According to the McDonald criteria	Healthy subjects	80/200	Age and sex	PCR and reverse hybridization	—	677 C/T; 1298 A/C	★★★★	MS
Gecene	2013	Turkey	Caucasian	A modified New York criteria for AS (1984)	Subjects with noninflammatory low back pain	50/50	Age, sex, and body mass index	Light Cycler real-time polymerase chain reaction	—	677 C/T	★★★★	AS
Huang	1997	Sweden	Caucasian	—	Healthy volunteers and healthy partners of patients	150/110	Ethnicity	PCR-RFLP	—	677 C/T	★★	MS
Izmirli	2016	Turkey	Caucasian	—	Psoriasis-free individuals	96/77	—	PCR-RFLP	—	677 C/T	★★	Psoriasis
Jin	2012	China	Asian	—	Subjects without any history and clinical evidence of autoimmune diseases	108/102	Age and sex	PCR-RFLP	—	677 C/T	★★★	Psoriasis
Karakus	2012	Turkey	Caucasian	The international criteria of BD for classification	Healthy subjects	318/207	Age and geographic area	PCR-RFLP	—	677 C/T	★★★★	BD
Kilic	2017	Turkey	Caucasian	—	Healthy subjects	84/212	Age and sex	Light cycler real-time PCR	—	677 C/T; 1298 A/C	★★★	Psoriasis
Kim	2013	South Korea	Asian	The criteria of the Behcet's research Committee of Japan	Healthy subjects unrelated to each other or to the patients	32/59	—	TaqMan	—	677 C/T	★★★	BD
Klotz	2010	Switzerland	Caucasian	According to the McDonald criteria	Healthy subjects	138/138	Age and sex	PCR-RFLP	—	677 C/T; 1298 A/C	★★★★	MS
Koubaa	2008	Tunisia	Caucasian	The criteria of the International Study Group for BD	Healthy volunteers	35/39	—	PCR-RFLP	—	677 C/T	★★★	BD
Lee	2016	Korea	Asian	The presence of hyperthyroidism, serum antithyroid-stimulating hormone receptor antibody (+), and/or a higher radioactive 131I uptake ratio with diffuse uptake.	Healthy subjects	50/100	—	PCR-RFLP	—	677 C/T; 1298 A/C	★★★★	GD
Liew	2012	Malaysia	Asian	According to clinical examination	Healthy subjects	200/167	Age, gender, and ethnicity	PCR-RFLP	—	677 C/T	★★★★★	Psoriasis
Luo	2018	China	Asian	Psoriasis Area and Severity Index	Healthy volunteers	420/424	Age and sex	PCR-RFLP	—	677 C/T; 1298 A/C	★★★★★	Psoriasis
Mao	2020	China	Asian	A modified New York criteria for AS (1984)	Healthy subjects	200/120	Age and sex	PCR-RFLP	—	677 C/T	★★★	AS
Mao	2010	China	Asian	The presence of hyperthyroidism, serum antithyroid-stimulating hormone receptor antibody (+), and/or a higher radioactive 132I uptake ratio with diffuse uptake.	Healthy subjects	199/235	—	PCR-RFLP	Genotyping was performed without knowledge of cases and controls, and repeated genotyping was used.	677 C/T; 1298 A/C	★★★	GD
Messedi	2013	Tunisia	Caucasian	The criteria of the International Study Group for BD	Healthy subjects	142/172	Age and sex	PCR-RFLP	—	677 C/T; 1298 A/C	★★★	BD
Naghibalhossaini	2015	Iran	Caucasian	According to the McDonald criteria	Healthy subjects	180/231	Age, gender and ethnicity	Mutagenically separated PCR and PCR-RFLP	—	677 C/T; 1298 A/C	★★★	MS
Ozkul	2005	Turkey	Caucasian	The criteria of the International Study Group for BD	Healthy subjects	59/42	Age and sex	PCR-RFLP	—	677 C/T	★★★	BD
Pi	2014	China	Asian	—	Healthy subjects	120/100	—	PCR-RFLP	—	677 C/T	★★	Psoriasis
Ricart	2006	Spain	Caucasian	The criteria of the International Study Group for BD	Healthy subjects	79/84	Age and sex	PCR-RFLP	—	677 C/T	★★★★★	BD
Szvetko	2007	Australia	Caucasian	—	Healthy subjects	140/140	Age, gender, and ethnicity	PCR-RFLP	—	1298 A/C	★★	MS
Tajouri	2006	Australia	Caucasian	—	Healthy subjects	104/104	Age, gender, and ethnicity	PCR-RFLP	—	677 C/T	★★★	MS
Toydemir	2000	Turkey	Caucasian	The international criteria of BD for classification	Subjects without a history of venous or arterial thrombosis	60/100	—	PCR-RFLP	Positive and negative control were used.	677 C/T	★★★	BD
Vasku	2009	Czech	Caucasian	—	Healthy subjects	410/244	—	PCR-RFLP	—	677 C/T	★★	Psoriasis
Wang	2000	China	Asian	—	Healthy subjects	39/79	—	PCR-RFLP	—	677 C/T	★★	Psoriasis
Weger	2008	Austria	Caucasian	According to clinical findings	Subjects without any history and clinical evidence of psoriasis	310/247	Age and sex	TaqMan	—	677 C/T	★★★★	Psoriasis
Wu	2007	China	Asian	—	Healthy subjects	123/129	Age and sex	PCR-RFLP	—	677 C/T; 1298 A/C	★★	Psoriasis
Xu	2005	China	Asian	A New York criteria for AS (1980)	Healthy volunteers	60/62	—	PCR-RFLP	—	677 C/T	★★	AS
Xu	2016	China	Asian	A modified New York criteria for AS (1984)	Healthy subjects	113/120	Age and sex	PCR-RFLP	—	677 C/T; 1298 A/C	★★★★	AS
Yigit	2015	Turkey	Caucasian	A modified New York criteria for AS (7th edition)	Healthy subjects	122/150	Age and ethnicity	PCR-RFLP	—	677 C/T	★★★★	AS

PCR-RFLP: polymerase chain reaction–restriction fragment length polymorphism; MS: multiple sclerosis; GD: Graves' disease; BD: Behcet's disease; AS: ankylosing spondylitis.

**Table 2:** Meta-analysis of *MTHFR* 677 C/T polymorphism with the risk of autoimmune diseases.

Diseases	Variables	*n*	CT versus CC			TT versus CC			Dominant model			Recessive model	
			OR (95% CI)	*P*_*Q*_		OR (95% CI)	*P*_*Q*_		OR (95% CI)	*P*_*Q*_		OR (95% CI)	*P*_*Q*_
Psoriasis	Total	14	1.33 (0.88-2.00)	<0.001		1.67 (0.94-2.97)	<0.001		1.44 (0.94-2.20)	<0.001		1.57 (1.00-2.45)	<0.001
	Asian	6	0.85 (0.52-1.40)	<0.001		1.33 (0.65-2.74)	0.003		0.94 (0.56-1.58)	<0.001		1.53 (0.95-2.47)	0.07
	Caucasian	8	1.93 (1.01-3.69)	<0.001		2.43 (0.92-6.40)	<0.001		2.06 (1.04-4.05)	<0.001		1.91 (0.84-4.32)	<0.001
	Study quality												
	High	5	1.41 (0.96-2.06)	0.003		2.73 (1.00-7.48)	0.008		1.51 (0.99-2.29)	<0.001		2.34 (0.98-5.58)	0.03
	Low	9	1.34 (0.69-2.61)	<0.001		1.34 (0.67-2.68)	<0.001		1.46 (0.74-2.86)	<0.001		1.33 (0.78-2.27)	0.003
BD	Total	10	1.05 (0.85-1.30)	0.21		2.00 (1.30-3.07)	0.11		1.06 (0.78-1.43)	0.09		1.97 (1.31-2.97)	0.12
	Caucasian	9	1.07 (0.86-1.34)	0.20		1.82 (0.83-4.00)	0.07		1.06 (0.77-1.46)	0.07		1.84 (1.19-2.86)	0.10
	Study quality												
	High	4	0.85 (0.46-1.56)	0.09		—	—		1.09 (0.82-1.45)	0.30		—	—
	Low	6	1.01 (0.75-1.36)	0.37		1.56 (0.97-2.52)	0.23		0.86 (0.43-1.72)	0.04		1.62 (1.03-2.54)	0.20
MS	Total	9	1.25 (0.89-1.75)	<0.001		1.69 (1.00-2.84)	0.004		1.33 (0.94-1.89)	<0.001		1.57 (1.03-2.38)	0.05
	Study quality												
	High	4	1.34 (0.91-1.98)	0.05		1.22 (0.76-1.96)	0.21		1.32 (0.90-1.92)	0.05		1.08 (0.69-1.71)	0.25
	Low	5	1.17 (0.66-2.09)	<0.001		2.18 (1.04-4.55)	0.008		1.33 (0.72-2.46)	<0.001		2.21 (1.53-3.19)	0.14
AS	Total	5	1.00 (0.76-1.32)	0.55		3.09 (1.99-4.80)	0.57		1.33 (1.04-1.72)	0.19		2.90 (1.92-4.38)	0.51
	Asian	3	1.16 (0.81-1.66)	0.90		2.91 (1.82-4.65)	0.50		1.60 (1.16-2.19)	0.45		2.67 (1.73-4.14)	0.44
	Caucasian	2	0.80 (0.51-1.25)	0.27		4.55 (1.27-16.27)	0.25		0.96 (0.63-1.48)	0.28		5.14 (1.44-18.33)	0.31
	Study quality												
	High	3	0.90 (0.63-1.29)	0.37		2.61 (1.42-4.82)	0.36		1.11 (0.79-1.55)	0.33		2.48 (1.42-4.32)	0.31
	Low	2	1.18 (0.76-1.85)	0.67		3.65 (1.94-6.90)	0.72		1.72 (1.16-2.53)	0.27		3.45 (1.86-6.42)	0.68
GD	Total	3	1.03 (0.43-2.47)	0.003		1.45 (0.50-4.16)	0.004		1.15 (0.49-2.72)	0.002		1.42 (0.78-2.60)	0.07
	Study quality												
	Low	2	0.85 (0.27-2.71)	0.003		0.81 (0.52-1.27)	0.10		0.88 (0.31-2.47)	0.004		1.07 (0.75-1.53)	0.94

MTHFR: methylenetetrahydrofolate reductase; OR: odds ratio; CI: confidence interval; *P*_*Q*_: *Q*-statistic for heterogeneity test among studies; BD: Behcet's disease; MS: multiple sclerosis; AS: ankylosing spondylitis; GD: Graves' disease.

**Table 3:** Meta-analysis of *MTHFR* 1298 A/C polymorphism with the risk of autoimmune diseases.

Diseases	Variables	*n*	AC versus AA			CC versus AA			Dominant model			Recessive model	
			OR (95% CI)	*P*_*Q*_		OR (95% CI)	*P*_*Q*_		OR (95% CI)	*P*_*Q*_		OR (95% CI)	*P*_*Q*_
MS	Total	7	2.36 (1.29-4.30)	<0.001		1.48 (0.72-3.04)	<0.001		2.31 (1.24-4.29)	<0.001		1.08 (0.54-2.16)	<0.001
	Study quality												
	High	3	4.64 (1.08-19.88)	<0.001		3.04 (0.45-20.77)	0.001		4.42 (0.84-23.42)	<0.001		1.64 (0.30-8.83)	0.002
	Low	4	1.50 (1.05-2.15)	0.06		1.27 (0.55-2.91)	0.002		1.50 (1.09-2.07)	0.09		1.02 (0.44-2.37)	<0.001
Psoriasis	Total	5	1.96 (0.79-4.86)	<0.001		1.85 (0.54-6.38)	0.002		2.02 (0.80-5.12)	<0.001		1.60 (0.58-4.47)	0.02
	Asian	2	1.23 (0.56-2.72)	0.02		3.25 (1.68-6.31)	0.68		1.31 (0.57-2.97)	0.01		2.68 (1.39-5.16)	0.84
	Caucasian	3	3.29 (0.30-35.92)	<0.001		1.61 (0.23-11.58)	0.007		3.33 (0.30-36.50)	<0.001		1.30 (0.27-6.35)	0.03
	Study quality												
	Low	4	2.18 (0.50-9.49)	<0.001		1.57 (0.33-7.52)	0.02		2.23 (0.51-9.80)	<0.001		1.33 (0.37-4.79)	0.06
GD	Total	3	0.91 (0.65-1.26)	0.91		1.72 (0.56-5.23)	0.31		0.94 (0.68-1.30)	0.71		1.77 (0.58-5.38)	0.32
	Study quality												
	Low	2	0.93 (0.65-1.35)	0.88		2.46 (0.65-9.26)	0.28		0.99 (0.70-1.42)	0.66		2.50 (0.67-9.38)	0.29

MTHFR: methylenetetrahydrofolate reductase; OR: odds ratio; CI: confidence interval; *P*_*Q*_: *Q*-statistic for heterogeneity test among studies; MS: multiple sclerosis; GD: Graves' disease.

## Data Availability

All data used to support the findings of this study are included within the article.
